# miR-940 potentially promotes proliferation and metastasis of endometrial carcinoma through regulation of MRVI1

**DOI:** 10.1042/BSR20190077

**Published:** 2019-06-10

**Authors:** Zhan Zhou, Ya-Ping Xu, Li-Juan Wang, Yan Kong

**Affiliations:** Department of Gynecology, Shandong Provincial Third Hospital, Jinan 250031, P.R. China

**Keywords:** endometrial carcinoma, metastasis, miR-940, MRVI1, proliferation

## Abstract

The specific functions and clinical significance of miR-940 in endometrial carcinoma (EC) have not been studied. First, we assessed the expression of miR-940 and MRVI1 in EC tissues collected from The Cancer Genome Atlas (TCGA) database and EC cell lines. miR-940 was significantly overexpressed in EC tissues and cell lines, particularly in RL95-2 cells. Correlation analysis showed that miR-940 expression level was remarkably associated with age, grade, and death. Moreover, the overall survival (OS) rate in the miR-940 low expression group was higher, compared with miR-940 high expression group. Univariate and multivariate models demonstrated that miR-940 expression, stage, and age were predictive indicators of OS. Moreover, there was no significance of the proliferation ability among the three EC cell lines (RL95-2, ISK, and KLE). To reveal the biological roles of miR-940, we respectively transfected RL95-2 cells with miR-940 mimics, miR-940 inhibitors, and control to further investigate the cell proliferation ability, and migration as well as invasion potential of RL95-2 cells. The transfection of miR-940 mimics significantly increased the proliferation and migration/invasion ability of RL95-2 cells. MRVI1 was predicted to be a potential target of miR-940 by means of *in silico* analysis followed by validation using luciferase reporter assays. MRVI1 was correlated with good prognosis. Moreover, forced expression of MRVI1 in miR-940 mimic transfected cells abolished the facilitation of miR-940 on cell proliferation, migration, and invasion of RL95-2 and KLE cells. In conclusion, our study demonstrates that miR-940 might function as a reliable diagnostic and prognostic signature in EC.

## Introduction

Endometrial cancer (EC) is one of the most common reproductive system malignancies for females in the world, and the incidence of this disease is rapidly increasing in recent years [1]. Of note, increasing annual incidence rate of 3.7% has been reported in China [2]. As documented, the majority of EC patients have promising therapeutic results after standard surgery, chemotherapy, and radiotherapy [3], with the 5-year survival rate for early diagnosed EC patients of approximately 80% [4,5]. However, the prognosis of advanced-stage EC patients is still poor [6]. Hence, the lack of effective treatments calls for the need of developing novel and promising strategies for treating this disease.

MicroRNAs (miRNAs), a class of small non-coding RNAs, function as the regulators of gene expression through targeting mRNA in a specific sequence way, and their dysregulation is a common characteristic during the development of tumor [7,8]. Moreover, miRNAs modulate some cellular processes, including cell proliferation, apoptosis, and angiogenesis [9]. Growing evidence has suggested that the aberrant expression of miRNAs is closely linked to the onset and progression of diverse cancers, such as breast cancer, lung cancer, hepatocellular carcinoma, and EC [10–14]. Furthermore, the abnormal expression of miRNAs has been suggested to be connected with the clinical outcome of patients with cancer [15–17]. In particular, it has been indicated that miR-940 acts as an oncogene or tumor suppressor in cancers. For example, miR-940 has been demonstrated to promote cell migration and invasion in gastric cancer [18]. High expression of miR-940 has been reported to contribute to the progression of cervical cancer and to shorten overall survival (OS) in patients with cervical cancer [19]. Moreover, miR-940 has been demonstrated to inhibit the invasive ability of cells, and promote E-cadherin activation in prostate cancer [20]. Yuan et al. [21] have demonstrated that decreased miR-940 induces cell proliferation, and is relevant to the short survival time in the patients with hepatocellular carcinoma. Nevertheless, the expression of miR-940 and the patho-mechanisms through which miR-940 contributes to the diagnosis and prognosis of EC have not been reported. MRVI1 is implicated to be involved in calcium signaling [22]. Kim et al. [23] have demonstrated that up-regulated MRVI1 is linked to the poor prognosis in the patients of ovarian cancer. However, the significance of MRVI1 is not clear in the miR-940 regulatory network of EC.

Herein, our study, for the first time, investigated the biological roles, molecular mechanism, and clinical value of miR-940 in EC. As expected, miR-940 was found to be highly expressed in EC tissues from The Cancer Genome Atlas (TCGA) database and cell lines, particularly in RL95-2 cells. The survival curve exhibited that the OS rate in the miR-940 low expression group was higher, compared with miR-940 high expression group. Univariate and multivariate models demonstrated that miR-940 expression, stage, and age were predictive indicators of OS. Moreover, silence of miR-940 inhibited cell growth, repressed cell migration and invasion. Most importantly, we verified that miR-940 suppressed MRVI1 expression via targeting its 3′-UTR. MRVI1 was down-regulated in EC and was correlated with good prognosis. In addition, the enhancing effects of miR-940 up-regulation on cell proliferation, migration, and invasion were rescued via MRVI1 overexpression in EC cells (RL95-2 and KLE). These data provided a better understanding of the molecular mechanism of miR-940 in the initiation and progression of EC.

## Materials and methods

### *In silico* analysis

The miR-940 and MRVI1 expression data of EC were retrieved from TCGA database which included 546 EC carcinoma samples and 33 normal tissues. We used EdgeR package to detect the difference of miR-940 and MRVI1 expression level between EC and normal tissues. Then, OS analysis was carried out for these patients. Because these clinical data were downloaded from TCGA database, not by ourselves, the data and analysis of our study did not require further approval of ethics committee.

### Cell culture

Human EC cell lines including RL95-2, ISK, and KLE were purchased from the Cell Bank of Chinese Academy of Medical Sciences (Shanghai, China). The normal human endometrial stromal cell line ESC, as negative controls (NCs), was obtained from Procell Life Science and Technology Co., Ltd (Wuhan, China). Cells were incubated at 37°C, 5% CO_2_ atmosphere and cultivated in RPMI-1640 medium with 10% fetal bovine serum (FBS), 100 µ/ml penicillin, and 0.1 mg/ml streptomycin.

### Cell transfection

The EC cells were planted into a six-well plate and grown to 70–80% confluence. Then, (i) the NC; (ii) the miR-940 mimic (transfected with miR-940 mimic sequence), and; (iii) the miR-940 inhibitor (transfected using miR-940 inhibitor sequence to knockdown miR-940) were synthesized by GenePharma (Shanghai, China), and transfected into EC cells by means of Lipofectamine 2000 based on the manufacturer’s regulations (Invitrogen, U.S.A.). MRVI1 overexpression plasmid without the 3′-UTR (pcDNA3.1-MRVI1) and empty plasmid (pcDNA3.1) were received from Guangzhou RiboBio Co., Ltd. (Guangzhou, China). Transfection efficiency was measured using quantitative reverse transcription polymerase chain reaction (RT-qPCR) method.

### RNA extraction and RT-qPCR

First, TRIzol (Takara Biotechnology Inc., Dalian, China) was used to extract total RNA from the cultured cancer cells, and then the RNA was reversed to cDNA relying on a HiFiScript cDNA Synthesis kit (CwBio, Beijing, China). After that, the real-time data were recorded and analyzed based on RT-qPCR (ABI PRISM 7900, Applied Biosystems, Foster City, CA, U.S.A.) using SYBR Green I (Roche Diagnostics, Mannheim, Germany). Next, 2^−ΔΔ*C*^_t_ method was applied to calculate the quantitative results. The relative expression level of miR-940 was quantitated relative to the level of the internal reference U6. The relative expression level of MRVI1 was quantitated to the expression level of the control GAPDH.

Primer sequences were:

miR-940: F-5′-ACACTCCAGCTGGGAAGGCAGGGCCCCCG-3′

R-5′-TGGTGTCGTGGAGTCG-3′

U6: F-5′-CTCGCTTCGGCAGCACA -3′

R-5′-AACGCTTCACGAATTTGCGT -3′

MRVI1: F-5′-CTCCGGTGTTGATGCAAACTC-3′

R-5′-GTCCCAAGCTGGGTTCCATT-3′

GAPDH: F-5′-GGAGCGAGATCCCTCCAAAAT -3′

R-5′-GGCTGTTGTCATACTTCTCATGG-3′

### Western blotting analysis

SDS/PAGE gel was employed to separate the proteins, and then these proteins were transferred to PVDF membranes (Bio-Rad, Hercules, U.S.A.). Subsequently, the membranes were incubated using primary antibodies (anti-MRVI1 (OriGene, at 1:5000 dilution) and anti-GAPDH (Santa Cruz Biotech, at 1:5000 dilution)) overnight at 4°C. After washing using TBST for three times, the membranes were incubated with HRP–conjugated secondary antibodies (Santa Cruz Biotech, at 1:5000 dilution). The protein bands were captured by chemiluminescence detection using ECL plus Western blotting detection kit (Thermo Fisher Scientific, U.S.A.). Then, the densitometry was used to analyze the density of the bands using Quantity One software (version 4.6.9, Bio-Rad, Hercules, CA, U.S.A.). GAPDH was used as the control.

### *In silico* target prediction and dual-luciferase reporter assay

The potential targets of miR-940 were predicted based on the online softwares TargetScan, miRanda, miRWalk, and miRDB. Finally, MRVI1 was predicted as a target gene of miR-940.

The relationship between miR-940 and MRVI1 was verified using the dual luciferase reporter assay. Wild-type (Wt) MRVI1 3′-UTR and mutated (Mut) MRVI13′-UTR were synthesized and cloned into the pMIR-REPORT luciferase plasmid. The HEK-293T cells at the logarithmic growth phase were seeded into the 96-well plate. After that, the cells were transfected by miR-940 mimics or miR-NC, combined with pMIR-MRVI1-3-UTR Wt or pMIR-MRVI1-3-UTR Mut using Lipofectamine 2000. After 48 h, the luciferase activity was obtained relying on the dual-luciferase reporter assay system (Promega, U.S.A.).

### Cell proliferation assay

Cell counting kit-8 (CCK-8) assay was implemented to investigate the proliferation ability of EC cell lines (RL95-2, ISK, and KLE) and the normal human endometrial stromal cell line ESC. After RL95-2, ISK, KLE, and ESC cells were cultured into 96-well plates and cultivated in 5% CO_2_ at 37°C, CCK-8 solution was added in each well to measure the relative cell proliferation activity at 0, 24, 48, 78, and 96 h after culture. The absorbance at 450 nm was monitored using a microplate reader.

Moreover, CCK-8 assay was implemented to investigate the effect of miR-940 on the proliferation ability of EC cells. In detail, EC cell suspension was seeded into 96-well plates and incubated at 37°C and 5% CO_2_. After RL95-2 cells were transfected with miR-940 mimics, miR-940 inhibitors, or control, CCK-8 solution was added in each well to measure the relative cell proliferation activity at 0, 24, 48, 78, and 96 h post-transfection. The absorbance at 450 nm was monitored using a microplate reader. GraphPad Prism 5 was utilized to generate the proliferation curves. The relative cell proliferation capacity was normalized to the proliferation activity of RL95-2 cells in the control group. The *t* test was used to compare the differences in cell growth between the transfection group and control group. All experiments were repeated three times.

### Wound-healing assay

This assay was utilized to detect the migration ability of EC cells. In detail, a pipet tip was used to make a scratch in a monolayer of transfected cells. Fresh medium was put into the plates immediately to discard the floating cells, and we recorded the scratch and surrounding cells after scratching. Then, photographs (at ×100 magnification) were captured at 24 h to determine the wound closure using microscope (Olympus, Tokyo, Japan). Migration ability was defined as a ratio of the area covered by the cancer cells, relative to the initial wound area. Each assay was performed in triplicate. Statistical Product and Service Solutions (SPSS) 22.0 software was used for data analysis.

### Invasion assay

Invasion assay was conducted in chamber of 8-mm Transwell inserts with Matrigel. EC cells were added to the top chamber of each insert in serum-free medium (1:6), and serum medium was utilized in the lower chamber as the attractant. Migrated cells were fixed using 4% paraformaldehyde for 30 min and stained in dye solution including 0.1% Crystal Violet for 20 min. The migrated cells with magnification (100×) were counted and photographed based on an inverted microscope (Olympus, Tokyo, Japan). Each assay was repeated three times independently. SPSS 22.0 software was used for data analysis.

### Statistical analysis

SPSS 22.0 software was utilized to perform the data analysis. The data were expressed in the form of mean ± standard deviation (SD). The differences of two groups were compared relying on *t* test, and one-way analysis of variance (ANOVA) test followed by Student–Newman–Keuls test was used to compare the parameters of multi-groups based on univariate. Kaplan–Meier method was used to construct survival curves on the basis of the miR-940 and MRVI1 expression level, and log-rank test was applied to investigate the survival differences. Univariate and multivariate Cox regression models were used to evaluate the prognostic role of miR-940 in EC patients. *P*<0.05 was defined as the statistical significance.

## Results

### miR-940 is highly expressed in EC tissues and cell lines

With the goal of clarifying the biological functions of miR-940 in EC, we investigated the expression of miR-940 in 546 EC tissue specimens and 33 normal specimens obtained from TCGA database. We found that the miR-940 was remarkably up-regulated in EC tissues, relative to normal samples (*P*<0.001; Figure 1A). To confirm this result based on the bioinformatics analysis, we subsequently detected the expression level of miR-940 in three EC cell lines (RL95-2, ISK, and KLE) and one normal cell (ESC). In line with the results in EC tissues, miR-940 levels were significantly higher in all EC cell lines than that in ESC cells (*P*<0.001; Figure 1C). These demonstrate that miR-940 might function as an oncogene in EC progression.

**Figure 1:** miR-940 is enhanced in EC, and linked to poor prognosis (**A**) Expression of miR-940 in 546 EC patients and 33 normal individuals. The miR-940 expression level was significantly increased in EC patients compared with the normals. (**B**) Kaplan–Meier survival curves showed that the OS was worse in the patients with high miR-940 expression, relative to low miR-940 expression. **P<0.001. (**C**) Expression of miR-940 in the EC cell lines (RL95-2, ISK, and KLE) and one normal cell (ESC). miR-940 levels were significantly higher in all EC cell lines than that in ESC cells. (**D**) CCK-8 assay was used to investigate the growth ability of EC cell lines (RL95-2, ISK, and KLE) and the normal human endometrial stromal cell line ESC. The results showed that RL95-2 cells had the strongest proliferation ability at 48, 72, and 96 h compared with other cells, but there was the lowest growth capacity of KLE cells among the three EC cells. **P<0.001.

### Connection of miR-940 expression level with the clinical parameters in EC

On the basis of the median value of miR-940 expression level, the EC patients were classified into an miR-940 low expression group and an miR-940 high expression group. Clinical parameters including age, grade, histological type, stage, and death were compared in these two groups (Table 1). From this table, we found that the miR-940 expression level was remarkably linked to age, grade, and death (*P*<0.05). Nevertheless, there was no association between the miR-940 expression and other parameters including histological type, and stage (*P*>0.05).

**Table 1:** Correlation between miR-940 expression and clinicopathological parameters of EC

Characteristics	Expression of miR-940		*P*-value
	Low	High	
**Age**			0.002*
<60	81	52	
≥60	126	155	
**Grade**			0.000*
G1+G2	106	56	
G3	101	151	
**Histological_type**			0.289
Endometrioid endometrial adenocarcinoma	162	149	
Mixed serous and endometrioid	8	8	
Serous endometrial adenocarcinoma	37	50	
**Stage**			0.080
I+II	157	141	
III+IV	50	66	
**Death**			0.006*
No	183	162	
Yes	24	45	

^*^denotes the statistical difference.

### Survival and prognosis analysis for EC patients

The Kaplan–Meier survival curve for EC patients based on miR-940 expression level is shown in Figure 1B, which exhibited that the OS rate in the miR-940 low expression group was higher, compared with miR-940 high expression group (*P*<0.05). This result implies that high expression of miR-940 is correlated with poor prognosis.

Then, univariate and multivariate Cox regression models were used to evaluate the prognostic role of miR-940 in EC patients (Table 2). In the univariate analysis, we found that miR-940 expression, stage, histological type, age, and grade (*P*<0.05) were significantly associated with OS in EC patients. Among the multivariate analysis results, stage and age (*P*<0.05) were the predictive indicators of OS.

**Table 2:** Univariate and multivariate COX analyses of clinical prognostic factors of EC

Variables	Univariate analysis			Multivariate analysis		
	*P*-value	HR	95%CI	*P*-value	HR	95%CI
miR-940 expression	0.005*	2.033	1.238–3.337	0.131	1.479	0.890–2.459
Stage	0.000*	4.382	2.714–7.074	0.000*	3.849	2.333–6.348
Histological type	0.000*	1.699	1.329–2.172	0.465	1.110	0.840–1.466
Age	0.000*	3.526	1.748–7.112	0.002*	3.147	1.528–6.480
Grade	0.000*	2.935	1.630–5.283	0.225	1.512	0.775–2.952

Abbreviations: HR, hazard ratio; 95%CI, 95% confidence interval.

^*^stands for statistical difference.

### Transfection of miR-940 mimics or inhibitors promotes or inhibits cell proliferation

From Figure 1C, we found that miR-940 level was the highest in RL95-2 cells. Then, we used CCK-8 assay to investigate the growth ability of EC cell lines (RL95-2, ISK, and KLE) and the normal human endometrial stromal cell line ESC. Based on Figure 1D, we found that RL95-2 cells had the strongest proliferation ability at 48, 72, and 96 h compared with other cells, but there was the lowest growth capacity in KLE cells among the three EC cells. Of note, there was no significance of proliferation rate among these three EC cells. Thus, RL95-2 cells were selected and used to conduct the miR-940 transfection to further measure the biological roles of miR-940 for EC, and KLE cells were used to verify the biological functions of miR-940 in EC. The results of RT-qPCR experiments showed that the transfection of miR-940 mimics caused an up-regulation of miR-940, whereas the inhibitor suppressed the miR-940 expression effectively (*P*<0.001, Figure 2A). We then investigated the roles of miR-940 on the cell growth of RL95-2 cells at 24, 48, 72, and 96 h using CCK-8. The transfection of miR-940 mimics significantly increased the proliferation of RL95-2 cells, and the RL95-2 cell growth in the miR-940 inhibitor group was remarkably inhibited at 48, 72, and 96 h after transfection (Figure 2B).

**Figure 2:** miR-940 inhibits cell proliferation of EC cell line RL95-2 (**A**) miR-940 expression level was significantly increased after transfection with miR-940 mimics, while its level was remarkably decreased after transfection with miR-940 inhibitors. (**B**) CCK-8 assay exhibited that the transfection of miR-940 mimics or inhibitors significantly increased/decreased the proliferation of RL95-2 cells at 48, 72, and 96 h post-transfection. Each assay was performed in triplicate. *P<0.05 and **P<0.001.

### Transfection of miR-940 influences the migration and invasion of RL95-2 cells

To investigate the effect of miR-940 on the migration and invasion ability of RL95-2 cells, we implemented the wound-healing and transwell experiments. The findings are displayed in Figure 3. Figure 3A,B exhibited that RL95-2 cells with miR-940 overexpression showed a faster closing of the scratch compared with the control group, but inhibition of miR-940 blocked the migration of cells. There were similar results in the aspect of invasion. As shown in Figure 3C,D, miR-940 overexpression significantly facilitated the ability to invade, relative to control group. In contrast, the invasion capacity of cells transfected by miR-940 inhibitor was attenuated. These results demonstrate that miR-940 overexpression can significantly promote metastatic properties of EC cells.

**Figure 3:** Effect of miR-940 on cell migration and invasion (**A**,**B**) Wound healing assay showed that miR-940 mimics and inhibitors promoted and inhibited cell migration in RL95-2 cells, respectively. (**C**,**D**) Transwell experiment displayed miR-940 mimics and inhibitors respectively facilitated and blocked cell invasion in RL95-2 cells. Blue lines in the middle denote the width of wound, and blue lines at the bottom right stand for the magnification of the images. Each assay was performed in triplicate. **P<0.001. Magnification ×100. Bar = 200 μm.

### MRVI1 is targeted by miR-940

As our results demonstrate that miR-940 plays key roles in EC progression, the question how miR-940 exerts its functions in EC needs investigation. In our study, bioinformatics algorithm was employed to predict the targets of miR-940. Finally, MRVI1 was identified as a direct target of miR-940 (context++ score from TargetScan).

With the goal of validating the bioinformatics result, luciferase reporter assay was performed to investigate the luciferase activity. The wild or mutant type of MRVI1-3′-UTR was established and inserted into the vector (Figure 4A). We observed that miR-940 mimics dramatically decreased the luciferase activity of pMIR-MRVI1-4-3-UTR (Wt) compared with the control (Figure 4B), whereas miR-940 did not impact the luciferase activity of the pMIR-MRVI1-4-3-UTR (Mut) group.

**Figure 4:** MRVI1 is a direct target of miR-940 (**A**) A binding site of miR-940 to MRVI1 3′ UTR and plasmids containing the MRVI1 3′UTR sequence. (**B**) miR-940 mimics dramatically decreased the luciferase activity of pMIR-MRVI1-4-3-UTR (Wt), while did not impact the luciferase activity of the pMIR-MRVI1-4-3-UTR (Mut) group. (**C**) Expression of MRVI1 mRNA was significantly increased in miR-940 mimics group, while it was down-regulated after transfected with miR-940 inhibitors. (**D**) Western blotting analysis of the expression of MRVI1 protein after transfection of miR-940. **P<0.001.

Next, in order to determine whether miR-940 influenced the expression of MRVI1, MRVI1 mRNA and protein expression in RL95-2 cells transfected with miR-940 mimic or miR-940 inhibitor were examined. Both mRNA (Figure 4C) and protein level (Figure 4D) of MRVI1 were decreased in the RL95-2 cells transfected by miR-940 mimic, but the opposite results were obtained in the miR-940 inhibitor group (Figure 4C,D). Overall, these indicate that miR-940 directly blocks MRVI1 expression.

### MRVI1 is down-regulated in EC and correlated with good prognosis

To further determine the association between MRVI1 and EC, we investigated the MRVI1 expression in 546 EC tissues and 35 normal tissues obtained from the TCGA database. The data demonstrated that MRVI1 was down-regulated in EC tissues compared with normal individuals (*P*<0.001, Figure 5A). According to the median value of MRVI1 expression, the EC patients were divided into MRVI1 low expression group or MRVI1 high expression group. The comparison of clinical factors (age, grade, histological type, stage, and death) in these two groups was performed (Table 3). On the basis of the comparison, we observed that the MRVI1 expression was strongly associated with age, grade, and death (*P*<0.05). No association was found between the MRVI1 expression and other clinical characteristics including histological type, and stage (*P*>0.05).

**Figure 5:** MRVI1 is decreased in EC, and linked to good prognosis (**A**) Expression of MRVI1 in 546 EC patients and 35 normal individuals. The MRVI1 expression level was significantly decreased in EC patients compared with the normals. (**B**) Kaplan–Meier curves show that high expression of MRVI1 had better prognosis than that of the low expression of MRVI1. **P<0.001.

**Table 3:** Relationship between MRVI1 expression and clinical characteristics in EC

Characteristics	Expression of MRVI1		*P*-value
	Low	High	
**Age**			0.012*
<60	54	78	
≥60	152	129	
**Grade**			0.004*
G1+G2	66	95	
G3	140	112	
**Histological_type**			0.200
Endometrioid endometrial adenocarcinoma	147	163	
Mixed serous and endometrioid	10	6	
Serous endometrial adenocarcinoma	49	38	
**Stage**			0.888
I+II	148	150	
III+IV	58	57	
**Death**			0.024*
No	163	181	
Yes	43	26	

^*^stands for the statistical difference.

Additionally, we examined the relationship between MRVI1 expression and OS. Kaplan–Meier curves revealed that high expression of MRVI1 had better prognosis than that of the low expression of MRVI1 (Figure 5B).

### MRVI1 overexpression obligates the effect of miR-940 on cells in RL95-2 and KLE cells

To further clarify whether MRVI1 was a functional target gene of miR-940 in the RL95-2 cells, MRVI1 overexpression was made in the RL95-2 cells which were transfected with miR-940 mimic. Based on the experiment results, we found that overexpressed MRVI1 rescued the suppressed expression of MRVI1 by miR-940 high expression (Figure 6A,B). As expected, MRVI1 overexpression abolished the facilitation of miR-940 on cell proliferation of RL95-2 cells (Figure 6C) and KLE cells (Figure 6D). The RL95-2 and KLE cell migration and invasion induced by miR-940 overexpression were also abolished after up-regulating MRVI1 (Figure 7). Collectively, these data suggest that miR-940 regulates RL95-2 and KLE cell proliferation and invasion through targeting MRVI1.

**Figure 6:** MRVI1 overexpression abolished the facilitation of miR-940 on cell proliferation of EC (**A**,**B**) Expression level of MRVI1 in miR-940 overexpression RL95-2 cells analyzed using Western blotting. (**C**) MRVI1 overexpression abolished the facilitation of miR-940 on cell proliferation of RL95-2 cells at 48, 72, and 96 h. *P<0.05 and **P<0.001. (**D**) MRVI1 overexpression abolished the facilitation of miR-940 on cell proliferation of KLE cells at 48, 72, and 96 h. *P<0.05 and **P<0.001.

**Figure 7:** The effect of MRVI1 up-regulation on the cell migaration and invasion of EC cells induced by miR-940 overexpression The cell migration of RL95-2 cells (**A**) and KLE cells (**B**) and invasion of RL95-2 cells (**C**) and KLE cells (**D**) induced by miR-940 overexpression was abolished after up-regulating MRVI1. **P<0.001.

## Discussion

The application of miRNAs has hold more attention for their diagnostic and prognosis in many human malignancies because of growing evidence suggesting their abnormal regulation in various cancers, including EC [24–26]. Nevertheless, the abnormal expression and potential functions of miR-940 in EC have not been investigated.

In our work, we observed that miR-940 was highly expressed in EC, and connected with poor prognosis of this cancer. To explore the roles of miR-940 in EC, miR-940 mimics or inhibitors were employed to increase or reduce miR-940 expression in RL95-2 cells. The results demonstrated that the transfection of miR-940 mimics significantly increased the proliferation and migration/invasion of RL95-2 cells, and the RL95-2 cell growth and migration/invasion in the miR-940 inhibitor group were inhibited, implicating that miR-940 might play an oncogene role in EC. Consistently, Fan et al. [27] have suggested that miR-940 induces the cell proliferation and migration of gastric cancer through up-regulating the expression level of programmed death ligand-1. Moreover, Liu et al. [18] have reported that miR-940 enhances the cell migration, invasion, and metastasis of gastric cancer via mediating the expression level of ZNF24. Another study has also demonstrated that high expression of miR-940 promotes proliferation of pancreatic cancer through regulating GSK3β and sFRP1 [28]. On the contrary, opposite findings were obtained. For example, Rajendiran et al. [20] have revealed that miR-940 attenuates growth ability, and suppresses the migratory and invasive potential of prostate cancer cells by regulating MIEN1. Ding et al. [29] have implied that miR-940 blocks cell migration and invasion via regulating CXCR2 in liver cancer. MiR-940 has also been demonstrated to inhibit pancreatic ductal adenocarcinoma growth through targeting MyD88 [30]. These discrepancies may indicate that miR-940 acts as different roles among diverse human cancers, partially through regulating different targets, to a certain degree.

MRVI1 was predicted to be the target of miR-940 and validated by luciferase report assay in the current study. MRVI1 has been demonstrated to participate in calcium signaling [22]. As reported, calcium signaling is known to play key roles in cancer progression, but also to exert crucial function in invasion and metastasis [31,32]. Kim et al. [23] have demonstrated that up-regulated MRVI1 is linked to the poor prognosis in the patients of ovarian cancer. Up to now, the relationship between MRVI1 and miR-940 in EC has been little noticed. In our work, we made an investigation of MRVI1 role in the proliferation and metastasis based on* in vitro* methods. After the RL95-2 and KLE cells were transfected by miR-940 mimics, MRVI1 expression level was reduced but the opposite results were found in the miR-940 inhibitor group. Importantly, MRVI1 overexpression abolished the facilitation of miR-940 on cell proliferation, migration, and invasion induced by miR-940 overexpression. These facts suggested that the inhibition roles of MRVI1 in the proliferation and metastasis might be mediated by miR-940. Collectively, the present work for the first time demonstrated that the metastasis ability of EC may be remarkably promoted by miR-940 transfection via regulating the MRVI1 expression.

In addition to the biological functions of miR-940 in EC, we also investigated its clinical significance. Several miRNAs including miR-200c-3p [33], miR-340 [34], and miR-181a [35] have been considered as signatures for EC patients. Understanding patho-mechanisms and target therapy in EC has benefited from these biomarkers. In the current study, the Kaplan–Meier analysis implied that the increased miR-940 expression was connected with worse OS for patients with EC. That is to way, up-regulation of miR-940 was associated with unsatisfied prognosis of EC.

Significantly, correlation analysis showed that miR-940 and MRVI1 levels were correlated with tumor grade but not stage in our study. A previous study has demonstrated that EC patients with nodal metastases are more likely to have higher tumor grades, and enhanced depth of invasion [36]. Moreover, Goh et al. [37] established a mouse model of breast cancer tumor formation and metastasis (MMTV-PyMT), and found that MMTV-PyMT mice exhibited a remarkable decrease in tumor grade (from high-grade to low-grade), and a significant inhibition in metastasis. Thus, miR-940 and MRVI1 levels correlating with tumor grade might be related to tumor metastatic potential.

## Conclusion

Taken together, we first reported miR-940 up-regulation in EC, and miR-940 functions as an oncogene in EC progression. Moreover, miR-940 overexpression serves as an indicator for poor prognosis. Mechanically, miR-940 decreases the expression of target gene MRVI1 which alleviates EC cell proliferation and invasion. Overall, this report could be a significant regulator–target combination to study and can be utilized as a prognostic indicator for EC. However, there were some disadvantages in the current study. To begin with, the relationship between miR-940/MRVI1 expression and OS was assessed based on the TCGA data, while this relationship lacks of confirmation using an* in vivo *animal model. Moreover, the biological roles of miR-940/MRVI1 axis in EC need to be verified using* in vivo* data from animal model in later work.

## Abbreviations

CCK-8: cell counting kit-8
CXCR2: CXC receptor 2
EC: endometrial carcinoma/cancer
GSK3β: glycogen synthase kinase-3β
HRP: horseradish peroxidase
MIEN1: migration and invasion enhancer 1
miRNA: microRNA
MRVI1: murine retrovirus integration site 1 homolog
MyD88: myeloid differentiation primary response gene 88
NC: negative control
OS: overall survival
PVDF: polyvinylidene fluoride
RPMI-1640: Roswell Park Memorial Institute-1640
RT-qPCR: quantitative reverse transcription polymerase chain reaction
sFRP1: secreted frizzled-related protein 1
SPSS: Statistical Product and Service Solutions
TBST: tris buffer saline Tween
TCGA: The Cancer Genome Atlas
ZNF24: Zinc finger protein 24
